The article "KIF3A and IL-4 are disease-specific biomarkers for psoriatic arthritis susceptibility" was published in 2017. Journal: Oncotarget.

# *KIF3A* and *IL-4* are disease-specific biomarkers for psoriatic arthritis susceptibility

**DOI:** 10.18632/oncotarget.20727

**Published:** 2017-09-08

**Authors:** Raffaella Cascella, Claudia Strafella, Michele Ragazzo, Laura Manzo, Gaetana Costanza, John Bowes, Ulrike Hüffmeier, Saverio Potenza, Federica Sangiuolo, André Reis, Anne Barton, Giuseppe Novelli, Augusto Orlandi, Emiliano Giardina

**Affiliations:** ^1^ Molecular Genetics Laboratory UILDM, Santa Lucia Foundation, Rome, Italy; ^2^ Department of Chemical Pharmaceutical and Biomolecular Technologies, Catholic University “Our Lady of Good Counsel” Laprakë, Rruga Dritan Hoxha, Tirana, Albania; ^3^ Department of Biomedicine and Prevention, “Tor Vergata” University, Rome, Italy; ^4^ Emotest Laboratory, Pozzuoli, Italy; ^5^ Department of Medical Science, Catholic University “Our Lady of Good Counsel” Laprakë, Rruga Dritan Hoxha, Tirana, Albania; ^6^ Anatomic Pathology, Department of Biomedicine and Prevention, Tor Vergata University of Rome, Rome, Italy; ^7^ Arthritis Research UK Centre for Genetics and Genomics, The University of Manchester, Manchester, UK; ^8^ Institute of Human Genetics, University of Erlangen-Nuremberg, Erlangen, Germany; ^9^ NIHR Manchester Musculoskeletal Biomedical Research Unit, Central Manchester Foundation Trust and University of Manchester, Manchester Academy of Health Sciences, Manchester, UK; ^10^ Anatomic Pathology, Department of Biomedicine and Prevention, Tor Vergata University of Rome, Italy, Tor Vergata University Hospital, Rome, Italy

**Keywords:** psoriatic arthritis, susceptibility, bone metabolism, 5q31 locus, linkage disequilibrium

## Abstract

To date, the genes associated with Psoriatic Arthritis (PsA) are principally involved in inflammation, immune response and epidermal differentiation, without any information about the relationship between disease and bone metabolism genes. Our work was focused on 5q31 locus, which contains several genetic variants significantly associated with PsA. The study involved 1526 subjects (500 PsA, 426 PsV, 600 controls). The region was evaluated by selecting and genotyping the SNPs of interest by Real Time PCR and direct sequencing. The results were subjected to biostatistic and bioinformatic analysis.

The case-control study highlighted a significant association between *KIF3A/IL-4* and PsA, but not with PsV (Psoriasis Vulgaris) patients. In addition, the haplotype analysis revealed two haplotypes significantly associated with PsA susceptibility. The Linkage Disequilibrium (LD) study showed the presence of a specific block in high LD within 132,692,628-132,737,638 bp of 5q31, giving additional evidence of specific association of the 5q31 region in PsA patients. Moreover, KIF3A expression was assessed by immunohistochemistry assays which showed a marked and significant difference of KIF3A expression between pathological and normal tissues. Our analysis described *KIF3A* and *IL-4* as novel susceptibility genes for PsA, suggesting a clear implication of bone metabolism genes in the disease etiopathogenesis.

The article "KIF3A and IL-4 are disease-specific biomarkers for psoriatic arthritis susceptibility" was published in 2017. Journal: Oncotarget.

## INTRODUCTION

Extensive research has been carried out in order to draw an exhaustive genomic picture of the etiopathology of Psoriatic Arthritis (PsA, OMIM #607507). Up to date, most of the knowledge concerning the etiopathogenetic mechanisms of PsA essentially refers to genes involved in inflammation, immune response and epidermal differentiation [1–3]. PsA is an inflammatory arthropathy caused by the erosion and inflammation of the distal joints (in particular the interphalangeal and sacroiliac joints) and the entheses (the insertion sites between the tendon and the bone) with a possible involvement of the axial skeleton. The disease can also be characterized by dysregulated bone formation at the level of the peripheral or axial skeleton. The degree of severity and the course of PsA are variable, ranging from mild to more severe forms, leading to a destructive and progressively debilitating course [4]. The prevalence of PsA is estimated to be 0.3%-1% in the general population, although it is often developed in combination with Psoriasis Vulgaris (PsV, OMIM #177900; in 20-30% of cases), and it presents an incidence peak between 20 and 40 years of age independent of gender [5–7].

Even though the pathogenetic molecular pathways are still unclear, the damage in PsA is known to be correlated to inflammatory events that enhance the production of inflammatory molecules and the activation of immune cells (T-cells). The migration of inflammatory molecules and T-cells to the synovia thereby disrupts the metabolic and remodelling (osteoblasts/osteoclasts differentiation) activities of the bone. This process finally results in the erosion, osteolysis and loss of Bone Mineral Density (BMD), which are responsible of the bone deformation and destruction in PsA [3]. Consequently, common symptoms of the disease are inflammation of the joints which become painful, stiff, swollen and hot.

PsA is classified as a multifactorial disease in which environmental and genetic factors are likely to influence susceptibility to the disease. Environmental factors include stress, low-humidity, drugs, smoking, obesity and chronic infections [7]. The genetic contribution has been extensively investigated through a number of studies (linkage analysis on twins and families, case-control studies, and genome-wide association studies). In fact, a recurrence risk of 40 has been reported among first-degree relatives of patients with PsA [1, 7]. Several susceptibility genes have been found to confer a higher risk for PsA (and PsV for most of them), such as *HLA* (Cw^*^06:02, B^*^08, B^*^27, B^*^38), *LCE3B*, *LCE3C*, *TRAF3IP2*, *ILs* (*IL-17*, *IL-23*, *IL-23R, IL12, IL12B, IL21*), *RUNX3*, *TNF-α, TNIP1, PTPN22, DENND1B, SLC22A5* [8–15]. As expected, all of the genes are involved in inflammatory, immunologic and epidermal differentiating mechanisms. However, information about the genes potentially implicated in the disruption of bone homoeostasis in PsA has yet to be clarified.

The article "KIF3A and IL-4 are disease-specific biomarkers for psoriatic arthritis susceptibility" was published in 2017. Journal: Oncotarget.

In this context, the investigation of such genes may reveal attractive insights into the principal mechanisms of the disease. Given these premises, we focused our attention on the 5q31 locus, which contains several genetic variants significantly associated with PsA [14, 16] as well as a number of genes (280, including *ADRB2*, *SPARC*, *TGFBI*, *IL-4*, *KIF3A*, *SMAD5*, *GDF9*, *PDLIM4*) involved in the osteogenic, differentiating and remodelling activities of the bone. Among them, *KIF3A* (*Kinesin Family Member 3A*) caught our attention as it was previously associated with other multifactorial disorders that share etiopathogenetic pathways similar to PsA. In fact, *KIF3A* has been associated with Atopic Eczema (AE), which is a chronic inflammatory skin disease characterized by a multifactorial inheritance pattern [17]. Genetic evidence highlighted the implication of genes involved in skin barrier dysfunction, excessive immune and inflammatory responses which are similar in PsA. *KIF3A* has a size of 47,986 bases and includes 17 exons and 20 introns. *KIF3A* codes for the homonymous protein (KIF3A) that is a member of the Kinesin family protein (a class of motor proteins involved in the intracellular transport). KIF3A is ubiquitously expressed in several tissues, such as nervous tissue, bone, skin, kidney. The protein takes part in several molecular pathways including skin homoeostasis and skeletal morphogenesis. Studies on *KIF3A* knock-out mice demonstrated that the gene ablation led to disruption of the normal skeletal development [18–20]. Given these data, *KIF3A* represents a good positional and functional candidate gene potentially involved in PsA etiopathogenesis. Thus, we decided to investigate the *KIF3A* gene and its flanking regions (132,692,628-132,737,638 bp) as a susceptibility locus in PsA.

## RESULTS

### Genetic studies

Our research work essentially explored 5q31 locus, with a particular focus on *KIF3A* gene and its flanking regions (132,692,628-132,737,638 bp). To this purpose, we performed an *in-silico* study of SNPs able to describe the maximum variability of the 5q31 genomic region of interest, paying attention to the frequency and the specific position of variants throughout the locus. The analysis led to the selection of four SNPs that are rs2227282 (C/G), rs2285700 (A/C), rs10062446 (A/T), and rs2897442 (A/G). However, a careful bioinformatic research indicated that rs2227282 was localized in the *IL-4* gene, while the rs2285700, rs10062446, and rs2897442 were positioned in the *KIF3A* gene (Table 1, Figure 1).

The article "KIF3A and IL-4 are disease-specific biomarkers for psoriatic arthritis susceptibility" was published in 2017. Journal: Oncotarget.

**Table 1:** The selected SNPs on genomic regions falling within 132,692,628-132,737,638 bp (5q31). (^*^): db SNP on NCBI Reference Assembly; (^#^): HapMap refSNP

SNPs	Position (^*^)	Gene (^*^)	Alleles (^#^)	Frequencies (^#^)
**rs2227282**	132.677.487	*IL-4*	C/G	G: 0.735; C: 0.265
**rs2285700**	132.703.440	*KIF3A*	A/C	A: 0.726; C: 0.274
**rs10062446**	132.704.682	*KIF3A*	A/T	A: 0.721; T: 0.279
**rs2897442**	132.713.335	*KIF3A*	A/G	A: 0.692; G: 0.308

**Figure 1:** Illustration of 5q31 locus, including the genes and the SNPs selected by *in-silico* analysis

The case-control study (1526 subjects, including 500 PsA, 426 PsV, 600 controls) revealed significant allele association with susceptibility to PsA (Table 2). In fact, the rs2227282 had a *p*=2.09601^*^10^-5^ and OR (G)=1.4 (95%CI: 1.12-1.73). The rs2285700 had a *p*=3^*^10^-3^ and OR (A)=1.3 (95%CI: 1.01-1.60). The rs10062446 had a *p*=5^*^10^-3^ and OR (A)=1.3 (95%CI: 1.0-1.57). The rs2897442 had *p*=1.2^*^10^-4^ and OR (A)=1.4 (95%CI: 1.09-1.71). Interestingly, the same SNPs were further genotyped in the cohort of PsV patients (n=426) without reporting a significant association. This result indicates that PsA and PsV are characterized by genetic signatures which confer specific susceptibility to develop one disease or another. Given these data, *IL-4* and *KIF3A* are genetically associated exclusively with PsA. The SNPs of interest are mapped within the intronic regions of the genes, and the prediction analysis for the impact of these SNPs did not reveal substantial alteration of the splice sites. This result suggested that the SNPs may have an impact on the proteins other than a change of splicing activity. Given the association of *IL-4* and *KIF3A* with PsA and their closeness within the 5q31 locus, we evaluated the Linkage Disequilibrium (LD) pattern in cases and control samples. The LD analysis was performed in order to further support our results and provide additional evidence of specific association of 5q31 with PsA. As expected, the LD patterns between the two groups were almost overlapping (D’=0.95) revealing two PsA-associated haplotypes, C-A-A-A with *p*=1.70652^*^10^-6^ and OR=1.6 (95%CI: 1.2-2.0) and G-C-T-G with *p*=1.70652^*^10^-6^ and OR=0.6 (95%CI: 0.5-0.8), covering up to 97% of the variability of 132,692,628-132,737,638 bp of the 5q31 locus. As expected, the risk haplotype (C-A-A-A) reported a higher frequency in cases than in control subjects, while the protective haplotype (G-C-T-G) was more frequent in control samples (Table 3). Successively, a wider investigation of *KIF3A* locus revealed two SNPs, rs2277065 (A/G) and rs2277066 (G/C), within the promoter region that were significantly associated with PsA. In particular, the rs2277065 reported a *p*=0.001 and OR (A)=1.70 (95%CI: 1.22-2.36) and the rs2277066 had a *p*=0.004 and OR=1.52 (95%CI: 1.14-2.04) (Table 4). In addition, we assessed the potential impact of the SNPs on the splicing activity through the bioinformatic prediction analysis which reported a potential alteration of splicing activities. As expected, the evaluation of the LD between rs2277065 and rs2277066 showed a D’=0.94 thereby showing a high LD. Given these results, we extended the LD analysis to the whole set of SNPs considered in this work (rs2227282, rs2285700, rs10062446, rs2897442, rs2277066 and rs2277065). The analysis reported a D’=0.79 in cases, while the control group showed a D’=0.18. On the basis of our results, we performed the haplotype analysis considering the SNPs of interest and obtaining several haplotype combinations. As shown in Table 5, 2 haplotypes resulted to be significantly associated with PsA, particularly: C-A-A-A-G-A reported a *p*=2.92^*^10^-7^ and OR=1.98 (95%CI: 1.52-2.59) while G-G-T-G-G-A had a *p*=3.8^*^10^-3^ and an OR=0.56 (95%CI: 0.41-0.75). These data suggested that the PsA susceptibility region is not localized within the promoter region; rather it can be specifically restricted to the *IL4*/*KIF3A* block. In particular, while the haplotype C-A-A-A-G-A (composed of risk alleles at *IL4/KIF3A* block and *KIF3A* promoter region) reported significant association values showing a risk effect on PsA susceptibility, the haplotype G-G-T-G-G-A (composed of protective alleles at *IL4/KIF3A* block and risk alleles at the *KIF3A* promoter region) showed a protective effect (Table 5).

The article "KIF3A and IL-4 are disease-specific biomarkers for psoriatic arthritis susceptibility" was published in 2017. Journal: Oncotarget.

**Table 2:** Case-control study performed on PsA and PsV patients

Disease	Locus	SNPs	AllelesFrequencies (C/Cn)	*p*	OR (95% CI)	Allele Effect
**PsA**	5q31	rs2227282	C:0.79/0.72	2.09601^*^10^-^	1.4 (1.12-1.73)	Risk
			G:0.21/0.28	^5^	0.7 (0.57-0.89)	Protective
	5q31	rs2285700	A:0.79/0.75	3^*^10^-3^	1.3 (0.51-1.60)	Risk
			C:0.21/0.25		0.8 (0.62-0.98)	Protective
	5q31	rs10062446	A:0.79/0.75	5^*^10^-3^	1.3 (1.0-1.57)	Risk
			T:0.21/0.25		0.8 (0.67-0.93)	Protective
	5q31	rs2897442	A:0.77/0.72	1.2^*^10^-4^	1.4 (1.09-1.71)	Risk
			G:0.23/0.28		0.7 (0.59-0.92)	Protective
**PsV**	5q31	rs2227282	C:0.69/0.72	ns	-	-
			G:0.31/0.28		-	-
	5q31	rs2285700	A:0.72/0.75	ns	-	-
			C:0.28/0.25		-	-
	5q31	rs10062446	A:0.72/0.75	ns	-	-
			T:0.28/0.25			
	5q31	rs2897442	A:0.74/0.72	ns	-	-
			G:0.26/0.28		-	-

**Table 3:** Haplotype analysis on *IL-4*/*KIF3A* block

Haplotypes	PsA patientsFrequencies	Control subjectsFrequencies	*p*	OR (95% CI)	Haplotype Effect
C-A-A-A	0.78	0.68	1.70652^*^10^-6^	1.6 (1.2-2.0)	Risk
G-A-A-A	0.02	0.01	ns	-	-
G-C-T-A	0.001	0.001	ns	-	-
C-C-A-G	0.001	-	ns	-	-
G-C-G-A	0.001	-	ns	-	-
C-C-T-G	0.013	0.01	ns	-	-
G-A-A-G	0.008	0.01	ns	-	-
G-A-T-G	0.006	-	ns	-	-
G-C-T-G	0.17	0.29	1.70652^*^10^-6^	0.6 (0.5-0.8)	Protective

Only the haplotypes with a frequency > 2% are reported.

**Table 4:** Case-control study performed on *KIF3A* promoter region in PsA patients

Disease	Locus	SNPs	Alleles	*p*	OR (95% CI)	Allele Effect
**PsA**	5q31	rs2277065	A	0.001	1.70 (1.22-2.36)	Risk
			G		0.59 (0.42-0.81)	Protective
	5q31	rs2277066	G	0.004	1.52 (1.14-2.04)	Risk
			C		0.65 (0.49-0.88)	Protective

**Table 5:** Haplotype analysis performed on *IL-4*/*KIF3A* block and *KIF3A* promoter region

Haplotypes	PsA patients Frequencies	Control subjects Frequencies	*p*	OR (95% CI)	Haplotype Effect
**C-A-A-A-G-A**	0.76	0.63	2.92^*^10^-7^	1.98 (1.52-2.59)	Risk
G-C-T-G**-G-A**	0.13	0.21	3.8^*^10^-3^	0.56 (0.41-0.75)	Protective
G-C-T-G-C-G	0.04	0.03	ns	-	-

The table shows only the haplotypes with a frequency > 2%. Risk alleles are written in bold characters.

### Immunohistochemical studies

Successively, we decided to assess the tissue localization of KIF3A through immunohistochemistry, in order to observe a differential expression of KIF3A in patients compared to control subjects. The immunohistochemical studies documented that KIF3A immunoreactivity was faint in tissue biopsies of normal synovial tissue (<25% positive cells on average, Figure 2a-2b), whereas KIF3A expression appeared more marked and present in more than 80% of positive cells on average in rheumatoid synovial tissue (Figure 2c-2d). Moreover, KIF3A expression was almost faint in macroscopically normal hip cartilage with less than 25% of positive cells on average (Figure 2e-2f), while KIF3A expression markedly increased (>80% positive cells on average; Figure 2g-2h) in hypertrophic chondrocytes from osteoarthritic cartilage. Semiquantitative evaluation confirmed the higher KIF3A expression in pathological compared to normal tissues (^**^p<0,007 and ^*^p<0,013, Figure 3). Altogether, the presented data highlights the potential involvement of a differential expression and function of particular bone-related genes (such as *KIF3A* and *IL-4*) in the etiopathogenesis of PsA.

The article "KIF3A and IL-4 are disease-specific biomarkers for psoriatic arthritis susceptibility" was published in 2017. Journal: Oncotarget.

**Figure 2:** KIF3A immunostaining of synovial and cartilaginous tissue Representative images of KIF3A immunostaining of osteoarthritic and rheumautoid synovial tissue **(a-d)** and macroscopically normal and osteoarthritic cartilage **(e-h)**. Diaminobenzidine as chromogen; original magnification: a, c, e and g at 100X; b, d, f and h at 400X. Abbreviations: normal synovial t.= normal synovial tissue; rheumatoid synovial t.= rheumatoid synovial tissue.

**Figure 3:** Semiquantitative evaluation of KIF3A immunostaining Bar graph showing the higher levels of KIF3A immunostainings in rheumatoid compared to normal synovial tissue (^**^p<0,007) and in osteoarthritic compared to normal hip cartilage (^*^p<0,013). Results are expressed as mean values± SEM.

## DISCUSSION

Among the connective tissues, the bone has one of the most dynamic metabolisms with constant turnover and remodelling activities. The homoeostasis between these two activities is maintained by the proper functioning of the osteoblasts (osteogenesis) and osteoclasts (bone resorption). In physiological conditions, bone homoeostasis is perfectly balanced and can promptly respond to different kinds of internal/external stimuli (mechanical stress, inflammation, trauma, bone regeneration). In the presence of PsA, the bone homoeostasis is heavily disrupted leading to bone erosion, structural alteration and new bone formation [21]. Moreover, patients with PsA often experience a BMD reduction that is responsible for the bone loss and increased predisposition to fractures [21–23]. However, the contribution of bone metabolism genes on the onset of PsA still remains unknown.

The results concerning the study of the 5q31 genomic regions falling within 132,692,628-132,737,638 bp in our cohort provided interesting insights into the potential involvement of bone-related genes in PsA etiopathogenesis. In fact, the strong genetic association of *KIF3A* and *IL-4* identified them as two novel susceptibility genes for PsA. Moreover, it is a matter of fact that the 5q31 locus, including both the genes, is known to be characterized by a complex LD pattern. As expected, the LD study of rs2227282, rs2285700, rs10062446 and rs2897442 in our PsA cohort reported a D’=0.95. This result indicates the presence of a specific block in high LD within 132,692,628-132,737,638 bp of 5q31, representing additional evidence of association of the 5q31 region in PsA patients. In fact, our previous study on 1962 PsA patients revealed association of rs715285 (A/G; located between *CSF2* and *P4HA2* genes, 132,149,690 bp) [14]. LD analysis (data not shown) confirmed the independence of the rs715285 signal from the *IL4*/*KIF3A* block (rs2227282, rs2285700, rs10062446 and rs2897442). Moreover, the analysis of the allele architecture revealed two associated-haplotypes with the same association degree (*p*=1.70652^*^10^-6^) but opposite effect on the susceptibility to PsA. In particular, the haplotype C-A-A-A was recognized to increase the risk for disease (OR=1.6) and was found more frequently in our patient cohort. On the other hand, the haplotype G-C-T-G was classified as protective for PsA (OR=0.6) and showed a higher frequency in our control subjects. Interestingly, both haplotypes cover the 97% of variability of the 5q31 region of interest. Successively, we extended our research to the *KIF3A* promoter region in order to detect variants that may influence or modify the transcriptional activity of the gene. On this subject, the rs2277065 and rs2277066 SNPs ended up to be associated with a higher susceptibility to PsA, as demonstrated by the significant association values (*p*=0.001 and OR=1.70; *p*=0.004 and OR=1.52, respectively). The association of both the SNPs with the disease was independent from the rs715285, as shown by the low LD among those polymorphisms (D’=0.10). Taken together, our results support the thesis that 5q31 is a locus specific for PsA. On this subject, it is important to remark that *KIF3A* and *IL-4* gave non-significant data from the genotyping/biostatistic analysis performed on our PsV cohort. The divergence of results between PsA and PsV samples may be linked to the molecular function displayed by the KIF3A and IL-4 proteins. In fact, both are known to take part in the modulation of osteogenic and remodelling activities of the bone at different levels. Several studies have demonstrated the role of IL-4 in the regulation of the osteoclastogenesis *in vitro* and *in vivo*. In particular, IL-4 showed to be able to prevent the differentiation of both the precursors and the mature osteoclasts by suppressing the expression of several modulators, such as RANKL, STAT6, NF-Kb and calcium signalling [24–26]. Concerning the role of KIF3A in the bone metabolism, recent research revealed that it participates in the commitment of osteoblast differentiation through a primary cilia induced-mechanism. This pathway was found to be activated in response to physical and mechanical stresses of the bone [27–29]. The mechanical loading plays a crucial role in bone remodelling and depends on external stimuli, such as ageing, weight, stress and trauma. In particular, mechanical stress and trauma have been supposed to be triggers of joint inflammation (especially enthesitis) and new bone formation in PsA and spondyloarthritis.

The article "KIF3A and IL-4 are disease-specific biomarkers for psoriatic arthritis susceptibility" was published in 2017. Journal: Oncotarget.

In fact, the lack of mechanical loading increases the turnover toward a more prevalent resorption activity, while the excessive mechanical loading damages the bone tissue and induces the remodelling [29–30]. The alteration of bone homoeostasis by excessive mechanical loading, damage and uncontrolled remodelling activity may thus contribute to the onset of arthropaties (osteoporosis, osteoarthritis, PsA) [21, 29–30]. Our results from the immunohistochemical studies clearly showed a marked and significant difference of KIF3A expression in rheumatoid and osteoarthritic tissue compared to normal synovial and cartilage tissues thus supporting the potential involvement of KIF3A in the etiopathogenesis of arthropaties. Unfortunately, any sinovial or cartilage tissue of patients with PsA were available for immunohistochemistry studies. These kind of samples are really difficult to find, although this will be certainly collected and analysed in the next future. Moreover, other studies are needed to investigate those KIF3A-dependent pathways which influence the maintenance of skin homoeostasis and skeletal morphogenesis. On the basis of these results, it would have been interesting to study the expression profile of the *KIF3A* gene in PsA patients with respect to control subjects. The gene is known to be highly expressed in the synovial tissue and, at very low levels, in the whole blood. Unfortunately, the expression analysis was not possible due to the lack of fresh synovial tissues from patients with PsA. It is important to remind that the collection procedure is highly invasive and painful for the patients and often disagree to donate a synovial tissue sample.

To date, the knowledge of PsA has been mainly concentrated on the research of genomic biomarkers and “molecular effectors” participating in immunologic, inflammatory and epidermal differentiation pathways leading to the onset and progression of disease. However, the role of bone metabolism and remodelling activities in PsA remains poorly understood. Few studies have tried to define which are the molecular players contributing to the disruption of bone homeostasis in PsA. The genomic features potentially linked with this process seem to be unexplored, since none of the genes controlling bone metabolism have been associated with the disease. In this context, we pointed our attention on *KIF3A* gene and its flanking regions (132,692,628-132,737,638 bp) considering its positional and functional properties potentially implicated in PsA. Our work revealed that *KIF3A* and *IL-4* are associated with PsA, indicating a clear implication of bone metabolism genes. These results pave the way for the characterization of a cluster of genes within the PsA-associated 5q31 locus in which immune/inflammatory and bone metabolism genes may actually interact in a unique etiopathogenetic pathway. In conclusion, the present data should be regarded as a starting point for future studies aimed to enrich the knowledge concerning 5q31 locus and its specific association with PsA, as well as the contribution of bone-related genes to the disease.

The article "KIF3A and IL-4 are disease-specific biomarkers for psoriatic arthritis susceptibility" was published in 2017. Journal: Oncotarget.

## MATERIALS AND METHODS

### Ethics statement

Investigation has been conducted in accordance with the ethical standards and according to the Declaration of Helsinki and according to national and international guidelines and has been approved by the authors’ institutional review board.

### Materials and methods

The main objective of the present study was the investigation of *KIF3A* gene and its flanking regions, in order to find evidence of potential connection between bone-related genes and PsA.

This study was designed as a case-control study involving a cohort of 1526 subjects recruited from “Tor Vergata” General Hospital in Rome. The cohort was subdivided in 500 patients affected with PsA, 426 patients affected with PsV and 600 healthy controls. The diagnosis of PsV and PsA were fulfilled according to the classical clinical criteria and the CASPAR Study Group criteria [31]. All patients were negative for the rheumatoid factor. Concerning the control subjects, they did not report evidence for PsV or PsA at the time of recruitment. Patients and control subjects have been recruited upon signature of informed consent. A blood sample was taken from all of the subjects in order to extract the genomic DNA. The DNA extraction was performed by the EZ1 Advanced XL automated extractor and the EZ1 DNA Blood 200 μl Kit (Qiagen).

The genomic variability of 5q31 locus was evaluated with special attention to the *KIF3A* gene and its flanking regions (132,692,628-132,737,638 bp). To this purpose, we first selected the SNPs that were able to represent the maximum variability of the region through the online tool “*HapMap3 Genome Browser release #2 (Phase 3-genotypes, frequencies & LD*)”. Afterwards, we chose the fewest number of SNPs able to characterize the maximum genomic variability of the 132,692,628-132,737,638 bp region (GRCh38). The SNPs were genotyped in all of the 1526 subjects in order to evaluate their association with PsA and PsV. The genotyping analysis was performed by TaqMan assays on a 7500 Fast Real Time PCR device (Applied Biosystems). Each Real Time PCR run was performed using a negative control and three positive control samples (homozygote wild-type, homozygote variant, heterozygote) which were previously confirmed by direct sequencing. The PCR sequence reactions were performed with BigDye Terminator v3.1 (Applied Biosystems) according to the manufacturer's instructions. After purification with BigDyeXTerminator (Applied Biosystems), samples were run on ABI3130xl (Applied Biosystems). The sequences were read by the Sequencing Analysis software v5.2 (Applied Biosystems).

The article "KIF3A and IL-4 are disease-specific biomarkers for psoriatic arthritis susceptibility" was published in 2017. Journal: Oncotarget.

The genotyping data obtained by Real Time PCR were interpreted using the Sequence Detection System 2.1 software (Applied Biosystems). In addition, the promoter region of *KIF3A* was initially resequenced in a small cohort of patients (n=50) in order to search for any variation that may alter the transcriptional profile of the gene in patients with PsA. Successively, the study of the *KIF3A* promoter region was extended to the whole study cohort through the genotyping analysis by TaqMan assays and Real Time PCR as previously described.

Concerning the evaluation of KIF3A expression on synovial and cartilage tissues, the traditional immunohistochemistry approach was adopted. Four-micrometer-thick serial sections were obtained from anonymised formalin-fixed, paraffin-embedded tissue samples (n=12) from Paraffin Block Archive of Anatomic Pathology of “Tor Vergata” University. Tissue samples included normal synovial tissue, normal hip, rheumatoid synovial tissue and osteoarthritic cartilage. Anonymised sections were stained with haematoxylin and eosin [32] for microscopic examination or employed for immunohistochemistry. For the latter, after deparaffinization and blocking of endogenous peroxidase activity with 0.2% H_2_O_2_ and heat-mediated antigen retrieval, sections were incubated with polyclonal rabbit anti-KIF3A (1:200, ABIN1387574, antibodies-online Inc.), followed by biotin-labelled goat anti-rabbit secondary antibody and streptavidin-horseradish peroxidase conjugated (1:100); 3,3-diaminobenzidine as final chromogen and haematoxylin as counterstaining were used [33]. All immunohistochemical procedures included internal positive and negative controls. KIF3A positivity was quantified using an arbitrary semiquantitative grading of the percentage of positive cells (0= 0%; 1= 0-25%; 2= 26-50%; 3=51-100%) from two researchers, with an intervariability <5% [34].

Genotyping results were subjected to biostatistical analysis in order to evaluate the association with PsV and PsA. First, the Hardy-Weinberg equilibrium was confirmed in each group of the cohort (PsA, PsV and control subjects). Afterwards, the association of the genotyped SNPs were measured by calculating the *p-value* (*p*) through a 2×2 contingency tables (http://www.physics.csbsju.edu/stats/contingency_NROW_NCOLUMN_form.html). The statistical associations were considered significant for *p*<0.05 with a 95% confidence interval. The strength of association was established by calculating the Odd Ratio (OR, http://www.hutchon.net/ConfidOR.htm).

The article "KIF3A and IL-4 are disease-specific biomarkers for psoriatic arthritis susceptibility" was published in 2017. Journal: Oncotarget.

Immunohistochemical data were analysed using Student's *t*-test. The results of semiquantitative evaluation were represented as the mean ± SEM. In general, *p*<0.05 was considered statistically significant. SPSS v16.0 (SPSS Incorporated) was used for statistical analyses.

The haplotype analysis was performed on the software UNPHASED version 3.1.7 (5/6/13) [35] and replicated on Haploview [36]. The evaluation of Linkage Disequilibrium for the SNPs of interest was assessed by the dedicated online tool (http://pharmgat.org/Tools/pbtoldplotform) and Haploview. Furthermore, the genotyping results were analysed by bioinformatic tools in order to characterize the SNPs (Single Nucleotide Polymorphisms) and the molecular function of the genes included in the region of interest (NCBI, HapMap, Ensembl, Genome Browser, GeneCards, 1000 Genome Browser). The polymorphisms were subjected to prediction analysis with the purpose of assessing any potential splice site variation (Mutation Taster and Human Splice Finder).

## Abbreviations

PsA: Psoriatic Arthritis
PsV: Psoriasis Vulgaris
KIF3A: Kinesin Family Member 3A
*p*: p-value
OR: Odd Ratio
LD: Linkage Disequilibrium
SNPs: Single Nucleotide Polymorphisms
BMD: Bone Mineral Density
